This article has been retracted.

# Oncological Effects and Prognostic Value of AMAP1 in Gastric Cancer

**DOI:** 10.3389/fgene.2021.675100

**Published:** 2021-06-17

**Authors:** Jiao Li, Shan Tian, Yingyun Guo, Weiguo Dong

**Affiliations:** ^1^Department of Gastroenterology, Renmin Hospital of Wuhan University, Wuhan University, Wuhan, China; ^2^Central Laboratory of Renmin Hospital, Wuhan, China; ^3^Key Laboratory of Hubei Province for Digestive System Disease, Wuhan, China

**Keywords:** AMAP1, gastric cancer, survival, biomarker, has-mir-192

## Abstract

**Purpose:**

We examined the diagnostic significance, prognostic value, and potential function of AMAP1 in gastric cancer (GC).

**Methods:**

Comprehensive bioinformatic analysis was conducted to investigate differential expression of AMAP1 mRNA and protein in GC. Meta-analyses were utilized to determine the overall prognostic correlation of AMAP1 mRNA in patients with GC. A panel of vitro assays was applied to assess target microRNA and AMAP1 protein in GC cell lines and tissues, respectively.

**Results:**

AMAP1 mRNA and protein levels were upregulated in GC specimens, compared to matched normal tissues. AMAP1 mRNA exhibited promising results regarding differential diagnosis of GC and normal tissue. Meta-analysis based on the TCGA and GEO databases revealed that high AMAP1 mRNA abundance was associated with poor overall survival (HR = 1.42; 95% CI: 1.06–1.89) and was correlated with reduced progression-free survival (HR = 1.89; 95% CI: 1.51–2.36) in GC patients. Moreover, AMAP1 was negatively correlated with miR-192-3p (*r* = −0.3843; *P* < 0.0001). A dual-luciferase assay revealed that miR-192-3p targeted AMAP1. Levels of miR-192-3p were significantly higher in GC tissues and GC cells than in normal tissues and cells. Moreover, AMAP1 silencing resulted in reduced GC proliferation, migration, and invasion.

**Conclusion:**

AMAP1 is a novel oncogene in GC and is negatively correlated with by miR-192-3p. AMAP1 may act as a diagnostic and prognostic marker of GC.

## Introduction

Gastric cancer (GC) is a major global health problem with nearly 800,000 GC-related deaths every year (Bray et al., 2018). GC is particularly prevalent in older people (over 60 years old), and it is equally common in males and females (Marques-Lespier et al., 2016). However, GC incidence varies considerably across geographic regions, which is highest in East Asia (Torre et al., 2015). Even though therapies combining surgical resection with systemic chemotherapy have been used successfully in GC patients, the long-term outcome of GC leaves much to be desired (Anderson et al., 2015). Novel molecular biomarkers are thus required to improve diagnostic accuracy and prognosis in GC patients.

ArfGAP with SH3 domain, ankyrin repeat and PH domain 1 (AMAP1), located at 8q24p, encodes the ADP-ribosylation factor (ARF) GTPase-activating protein (Roy et al., 2019). As a classical member of the ARF superfamily, AMAP1 exerts various biological effects including regulation of the actin cytoskeleton, integrin adhesion, and tumor invasion and metastasis (Gasilina et al., 2019). Recent studies showed that AMAP1 promotes cell proliferation and tumor invasion in several cancer cells including triple-negative breast cancer (He et al., 2020), ovarian cancer (Zhang et al., 2018), laryngeal squamous cell carcinoma (Li et al., 2014), colorectal cancer (Muller et al., 2010), and prostate cancer (Lin et al., 2008). However, the role of AMAP1 during GC has never been examined.

Currently, it is unknown whether AMAP1 affects development and metastasis of GC. We thus investigated the diagnostic and prognostic value of AMAP1 mRNA in GC patients. We used the Human Protein Atlas (HPA) database to assess differential expression of AMAP1 protein in GC and normal tissue. The LinkedOmics database was used to test whether AMAP1 expression was correlated with that of miR-192. Moreover, we examined protein expression of AMAP1 and miR-192-3p in GC tissues and cell lines and explored the effects of AMAP1 knockout on GC proliferation, migration, and invasion.

## Materials and Methods

### Analysis of Public Databases

Expression profiles of AMAP1 mRNA in different cancer types were investigated using the Gene Expression Profiling Interactive Analysis (Tang et al., 2017) (GEPIA)^1^. Oncomine^2^, the GEO database, and the UCSC webtool (Goldman et al., 2020)^3^ were searched to analyze differential expression of AMAP1 mRNA in GC tissues and normal specimens. A Kaplan-Meier plot webtool (Gyorffy et al., 2013)^4^ was used to assess the prognostic value of AMAP1 mRNA in GC. The Human Protein Altas (HPA) database^5^ was searched to investigate AMAP1 protein expression during GC. The LinkedOmics webpage (Vasaikar et al., 2018)^6^ was browsed for enrichment analysis and identification of microRNAs associated with AMAP1 during GC.

### Meta-Analysis

The PubMed, Web of Science, Cochrane and Embase databases were comprehensively retrieved to identify the previous studies regarding the correlation between AMAP1 and prognosis of GC. Combined HRs and 95% CIs were measured by the STATA 12.0 software to study the correlation of AMAP1 expression with prognosis of GC patients. The heterogeneity across different datasets was represented by I^2^ statistics and detected by the *Q*-test. A random-effects model would be selected for combination if obvious heterogeneity (I^2^ > 50%). On the contrary, a fixed-effects model would be employed when little heterogeneity exists (I^2^ ≤ 50%).

### Tissue Samples and Cell Lines

GC tissues and corresponding normal samples were collected from 10 patients who were treated at the Gastrointestinal Surgery Department of Renmin Hospital of Wuhan University, Wuhan, China. The following inclusion criteria were used: (1) patients pathologically confirmed with gastric cancer; (2) patients subjected to surgery; (3) patients aged 18–80 years. The following patients were excluded: (1) patients with other malignant tumors; (2) patients who underwent systemic chemotherapy or radiotherapy before surgery; (3) patients refusing to participate in this study. This study was approved by the Ethics Committee of Renmin Hospital of Wuhan University (No. WDRY2021-K002). Normal human gastric epithelium cells (GES-1) and cells of four GC cell lines (AGS, MGC-803, HGC-27, and SGC-7901) were obtained from the China Center for Type Culture Collection (Wuhan, China). The five cell types were grown in DMEM (HyClone) supplemented with 10% fetal bovine serum (Gibco, United States) under 5% CO_2_.

### Western Blotting

Total proteins from human tissues and cell lines were extracted, and protein concentrations were measured using a BCA kit (Beyotime, China). Proteins were subjected to SDS-PAGE, and then transferred to polyvinylidene difluoride membranes. The membranes were blocked with 5% BSA and incubated with primary antibody against AMAP1 (ab208170; Abcam) overnight at 4°C. Then, the membranes were incubated with the horseradish peroxidase conjugated secondary antibody (AS1107, ASPEN) at room temperature for 1 h.

### Cell Transfection

SiRNAs specifically against AMAP1 (si-ASAP1-#1, si-AMAP1-#2, and si-AMAP1-#3), siRNA scrambled control (si-NC), miR-192-3p-mimics, miR-192-3p-NC were purchased from RiboBio (Guangzhou, China). Gastric cells were plated in 6-well plates with a density of 10^6^ cells/well. Subsequently, gastric cell transfection with the oligonucleotides was conducted using Lipofectamine 2000 (Invitrogen, Carlsbad, CA, United States).

### RT-PCR

Real-time Polymerase Chain Reaction (RT-PCR) assay was conducted as previously illustrated (He et al., 2020). The primer sequences of human AMAP1 were: forward CAGCCGGCGCTTCCC, reverse ATCAGAAAACGACCGGG ACC, and the primer sequences of human miR-192-3p were: forward TGCTGCCAATTCCATAGGTC, reverse CTCAACTG GTGTCGTGGAGTC. GAPDH (forward: GGAGCGAGAT CCCTCCAAAAT, reverse: GGCTGTTGTCATACTTCTCATGG), and U6 (forward: CGCTTCGGCAGCACATATAC, reverse: TTCACGAATTTGCGTGTCAT) were selected as internal controls for AMAP1 and miR-192-3p, respectively. Relative AMAP1 mRNA or miR-192-3p levels after correction for GAPDH or U6 control mRNA were measured using the 2−ΔΔCT method.

### Dual-Luciferase Assay

The wild-type (WT) segment of the AMAP1 3′-UTR including the miR-192-3p-binding sequence was integrated into a pGL6-miR vector to produce AMAP1-WT. The target-binding sequence between AMAP1 and miR-192-3p was mutated, and the mutant-type (MUT) segment was integrated in a pGL6-miR vector to produce AMAP1-MUT. AMAP1-WT or AMAP1-MUT and miR-192-3p-mimics or miR-NC and the control vector (pRL-TK) were co-transfected into SGC-7901 cells using Lipofectamine 2000 (Thermo Fisher Scientific, Waltham, MA, United States). After 48 h, a dual-luciferase reporter gene detection system was used to determine its luciferase activity.

### Wound-Healing Assay

For cell motility assay, the gastric cancerous cell lines were cultured in six-well plates. A 200-μL pipette tip was used to create a single scratch wound, and the cell debris were washed with phosphate buffer saline. The pictures were immediately captured at 0 h and 48 h after wounding.

### CCK-8 Assay

Gastric cancerous cells intervened with Si-AMAP1 or Si-NC were seeded in 96-well plates. Ten μL CCK-8 reagent (C0038, Biyuntian biotechnology company) was added for 2-h incubation, and then the absorbance at 450 nm was measured via a microplate reader (Thermo Fisher Scientific, United States).

### Transwell Assay

Gastric cancerous cells intervened with Si-AMAP1 or Si-NC were seeded into transwell chambers (Corning, United States) coated or uncoated with Matrigel. Medium containing FBS in the lower chamber was used as the chemoattractant. The migrated cells were initially fixed in methanol and then stained with 0.5% crystal violet. Finally, the migrated or invaded cancer cells were counted with the aid of microscope.

### Statistical Analysis

The RNA-sequencing data were analyzed with SPSS software (version 20.0) and GraphPad Prism for Windows (version 6.0). AMAP1 mRNA was expressed as mean with standard deviation and detected with student *t*-test for the normal distribution. As levels of miR-192-3p were skew distribution, the relationship between miR-192-3p and clinical features were analyzed with non-parametric test. Receiver operating characteristic (ROC) analysis was utilized to assess the diagnostic value of AMAP1 mRNA in differentiating GC from the normal tissues. The survival analyses were represented with the Kaplan-Meier curves, and examined by the log-rank test. The association between AMAP1 and gene expression or MicroRNA was measured by Spearman’s correlation. Difference was regarded as significant with the associated *P*-value less than 0.05.

## Results

### AMAP1 mRNA Expression in GC and Normal Tissues

The GEPIA database was used to explore the differential expression of AMAP1 mRNA in various cancers and corresponding normal organs. Compared with normal tissues, AMAP1 mRNA was significantly upregulated in GC, esophageal cancer, head and neck tumors, and pancreatic cancer (Figure 1). By contrast, AMAP1 mRNA was showed low expression in lung adenocarcinoma, uterine corpus endometrial carcinoma, and testicular germ cell tumors.

**FIGURE 1:** The distribution of AMAP1 expression in various cancers. AMAP1mRNA expression distributed in a body map **(A)**. Dot plot of AMAP1expression profile across all tumor samples and paired normal **(B)**. Bar plot of AMAP1expression profile in various cancers and paired normal **(C)**.

We used the Oncomine database and the UCSC and GEO webtools to assess AMAP1 mRNA expression in GC and matched normal tissues. Compared to normal tissues, AMAP1 mRNA levels were upregulated in GC tissues, based on the TCGA-STAD (Figure 2A), GSE29272 (Figure 2B), Chen Gastric (Figure 2C), and Derric (Figure 2D) Gastric datasets. ROC analyses were used to assess differences in AMAP1 mRNA between GC and normal tissues, and AMAP1 mRNA showed promising diagnostic results (Figures 2E–H). AMAP1 mRNA showed the highest diagnostic potential to discriminate GC from normal tissues in the Derric Gastric dataset, as revealed by an AUC of 0.9973 (Supplementary Table 1). We also examined associations between AMAP1 mRNA and clinical parameters according to the TCGA-STAD dataset. High AMAP1 mRNA levels were significantly correlated with advanced T stage (*P* = 0.0022), N stage (*P* = 0.0154), TNM stage (*P* = 0.0007), and larger tumor size (*P* = 0.0382), whereas no correlation was observed with age (*P* = 0.2849), gender (*P* = 0.944), G stage (*P* = 0.2574), M stage (*P* = 0.8495), and tumor status (*P* = 0.1678; Figure 3).

**FIGURE 2:** The expression and diagnostic significance of AMAP1mRNA in gastric cancer. Levels of AMAP1mRNA are statistically higher in gastric tissues than that in normal stomach tissues in TCGA-STAD **(A)**, GSE29272 **(B)**, Chen Gastric **(C)**, and Derric Gastric **(D)** datasets. ROC curves of AMAP1mRNA for the identification of gastric cancer in TCGA-STAD **(E)**, GSE29272 **(F)**, Chen Gastric **(G)**, and Derric Gastric **(H)** datasets.

**FIGURE 3:** Association between AMAP1mRNA based on TCGA-STAD dataset and clinical characteristics, including age **(A)**, gender **(B)**, G stage **(C)**, T stage **(D)**, N stage **(E)**, M stage **(F)**, TNM stage **(G)**, tumor size **(H)**, and cancer status **(I)**.

### Prognostic Value of AMAP1 in GC Patients

A Kaplan-Meier plot webtool was used to assess the prognostic value of AMAP1 mRNA in GC patients. Those GC patients with AMAP1 mRNA overexpression showed reduced overall survival (OS) compared to patients with low AMAP1 expression, according to the TCGA-STAD dataset (HR = 1.47, 95% CI: 1.04–2.08; *P* = 0.029; Supplementary Figure 1). Using the GEO database, this association between AMAP1 mRNA overexpression and reduced OS occurred in datasets GSE 15459 (HR = 1.76; 95% CI: 1.16–2.67; *P* = 0.0067) and GSE62254 (HR = 1.85; 95% CI: 1.26–2.7; *P* = 0.0014), but did not occur in datasets GSE 14210 and GSE 29272. Similarly, progression-free survival (PFS) was reduced in GC patients with AMAP1 overexpression compared to those with low AMAP1 expression, according to the TCGA-STAD dataset (HR = 3.08; 95% CI: 1.29–7.39; *P* = 0.0078; Supplementary Figure 1). Using the GEO database, this association was also observed in datasets GSE 14120 (HR = 1.77; 95% CI: 1.16–2.69; *P* = 0.0074), GSE 15459 (HR = 1.73; 95% CI: 1.13–2.63; *P* = 0.0099), and GSE 62254 (HR = 1.94; 95% CI: 1.34–2.82; *P* = 0.00037).

Meta-analyses were carried out to determine the correlation of AMAP1 mRNA overexpression and survival in GC patients. As no published references regarding the prognostic value of AMAP1 in GC patients were available, we only included results based on TCGA-STAD and GEO datasets. The overall HR of the correlation between overexpression of AMAP1 mRNA and OS was 1.42 (95% CI: 1.06–1.89; Figure 4A). Similarly, the pooled HR of the correlation of AMAP1 overexpression and PFS was 1.89 (95% CI: 1.51–2.36; Figure 4B). Based on the meta-analysis results, we could conclude that AMAP1 mRNA overexpression is correlated with inferior OS and reduced PFS in GC patients.

**FIGURE 4:** Forest plot of overexpression of AMAP1mRNA associated with poor survival in gastric cancer patients. Overall survival **(A)**, Progression-free survival **(B)**.

### AMAP1 Protein Expression During GC

The HPA database was searched to assess AMAP1 protein expression in several tumors, and AMAP1 protein levels were high in gliomas, GC, and prostate cancer, and they were low in skin and renal cancer (Figure 5A). Among 20 cases of GC tissues from 11 patients examined using immunohistochemistry (IHC), 15 cases showed strong staining, 4 case showed moderate staining, and 1 case showed low staining of AMAP1 protein; 2 normal gastric tissues showed low AMAP1 protein staining. Representative images of IHC staining from normal and GC tissues are shown in Figures 5B–E.

**FIGURE 5:** Expression of AMAP1 protein in cancer tissues. The differential expression of AMAP1 protein in various cancers **(A)**. Representative immunohistochemistry figures of AMAP1 protein in normal stomach specimens **(B,C)** and in GC tissues **(D,E)**.

### Biological and KEGG Pathways of AMAP1 in GC

In total, 14,491 genes associated with AMAP1 expression (*P* < 0.05) in 415 samples from the TCGA-STAD dataset were identified using the Linkedomics database (Supplementary Figure 2A). The top 50 genes that were positively and negatively correlated with AMAP1 in GC tissues are shown in Supplementary Figures 2B,C, respectively. To delve into the possible mechanisms of AMAP1 in GC, we performed enrichment analysis on AMAP1 co-expressing genes using the WEB-based GEne SeT AnaLysis Toolkit (Liao et al., 2019)^7^. Gene ontology (GO) analyses revealed that genes co-expressed with AMAP1 were mainly enriched regarding biological processes such as cell-cell adhesion through plasma-membrane adhesion molecules, regulation of trans-synaptic signaling, cell-substrate adhesion, synapse organization, axon development, and ribonucleoprotein complex biogenesis (Supplementary Figure 2D). KEGG analysis demonstrated that genes co-expressed with AMAP1 in GC were involved in various important signaling pathways, including focal adhesion, axon guidance, and cell adhesion molecules (Supplementary Figure 2E). A detailed description of GO and KEGG analysis results is shown in Supplementary Tables 2, 3, respectively.

### Association of AMAP1 With miR-192

MicroRNAs that were significantly associated with AMAP1 expression in 415 GC patients are shown in Figure 6A. The top 50 microRNAs that were positively and negatively correlated with AMAP1 in GC tissues are shown in Figures 6B,C, respectively. Among the top three microRNAs negatively associated with AMAP1 expression, only miR-192 was significantly correlated with AMAP1 expression, as revealed using the Targetscan and MiRDB webtools. A negative correlation of AMAP1 expression and miR-192 was observed (*r* = −0.3843; *P* = 1.821 × e-14; Figure 6D). Statistical analyses demonstrated that miR-192 expression was significantly correlated with the histological type of GC (Figure 6E), race (Figure 6F), and pathological T stage (Figure 6G). Detailed results regarding associations of miR-192 and critical clinical features are shown in Supplementary Table 4. A Kaplan-Meier plot webtool was used to explore the prognostic value of miR-192 in GC patients, showing that those with high miR-192 levels showed increased OS than patients with low miR-192 levels (HR = 0.62; 95% CI: 0.46–0.84; *P* = 0.0016; Figure 6H).

**FIGURE 6:** Identification of MicroRNAs associated with AMAP1mRNA expression in 415 gastric cancer samples from the linkedomics database. Volcano plot of MicroRNAs significantly associated with AMAP1mRNA **(A)**. The top 50 MicroRNAs positively correlated to the expression of AMAP1mRNA **(B)**. The top 50 MicroRNAs negatively correlated to the expression of AMAP1mRNA **(C)**. Scatter plot of the association between AMAP1mRNA expression and has-mir-192 **(D)**. Expression of hsa-miR-192 is associated with histological type **(E)**, race **(F)**, and T stage **(G)**. High levels of has-mir-192 predict favorable overall survival in gastric cancer patients **(H)**.

### Validation Using Vitro Experiments

Western blotting was performed to examine AMAP1 protein expression in normal and GC tissues, and AMAP1 protein was increased in all 10 GC tissues, compared with the corresponding paracancerous samples (Figure 7A). Moreover, AMAP1 protein levels measured by western blotting were substantially higher in GC cells of AGS, MGC-803, HGC-27, SGC-7901 cell lines than in GES-1 cells (Figures 7B,C). RT-PCR was performed to measure expression of miR-192-3p in tissues and GC cells. Levels of miR-192-3p were significantly upregulated in in GES-1, compared to the levels in the four types of GC cells (Figure 7D). As shown in Figure 7E, miR-192-3p was decreased in all 10 GC tissues, compared with the corresponding paracancerous samples.

**FIGURE 7:** Expression of AMAP1 protein and miR-192-3p in human tissues and cell lines. **(A)** AMAP1 protein was increased in gastric cancerous specimens compared with the matched normal tissues by western blot. **(B)** AMAP1 protein was up-regulated in gastric cancerous cell lines compared with GES-1 by western blot. **(C)** Quantitative analysis of AMAP1protein in cancerous and normal gastric cell lines. **(D)** Expression of miR-192-3p was lower in gastric cancer cell lines than GES-1 by RT-PCR. **(E)** Expression of miR-192-3p was down-regulated in gastric cancerous specimens compared to the matched normal tissues by RT-PCR. *P < 0.05.

The potential binding sequence between AMAP1 and miR-192-3p is listed in Figure 8A. We conducted a dual-luciferase reporter gene assay to determine whether miR-192-3p targeted AMAP1, as indicated by bioinformatic analyses. As shown in Figure 8B, miR-192-3p overexpression by mimics markedly reduced luciferase activity in AMAP1-WT HGC-7901 cells, whereas in AMAP1-MUT cells, it remained unchanged. When miR-192-3p was overexpressed by miR-192-3p-mimics in SGC-7901 and AGS cells, AMAP1 expression was substantially lower than in the control cells (Figure 8C).

**FIGURE 8:** AMAP1 is the target of miR-192-3p. **(A)** The potential binding sequence between AMAP1 and miR-192-3p. **(B)** Dual-luciferase reporter gene assay reveals that AMAP1 is the binding target of miR-192-3p. **(C)** Western blot was applied to detect the expression of AMAP1 protein in HGC-7901 and AGS cells transfected with miR-192-3p mimics or miR-192-3p -NC or control. **P < 0.01.

In order to examine the potential role of AMAP1 in GC, we knocked out AMAP1 expression in SGC-7901 cells. The relative levels of AMAP1 mRNA were lower in GC cells transfected with Si-AMAP1#1 than GC cells transfected with Si-AMAP1#2 (Si-AMAP1#1 vs. Si-AMAP1#2, *P* = 0.0198) or Si-AMAP1#3 (Si-AMAP1#1 vs. Si-AMAP1#3, *P* = 0.0297). So, Si-AMAP1-#1 was used for subsequent experiments due to its high efficiency (Supplementary Figure 3). Compared with the SGC-7901 cells interfered with Si-NC, those interfered with Si-AMAP1 showed lower rates of cell proliferation, as revealed by a CCK-8 assay (69.88 ± 5.49% vs. 100.00 ± 6.185%; *P* < 0.0001; Figure 9A). A wound-healing assay was used to assess invasion ability of SGC-7901 cells interfered with Si-AMAP1, showing that the rate of wound healing was lower, compared with gastric cells intervened with Si-NC (36.04 ± 2.79% vs. 56.69 ± 2.1%; *P* < 0.0001; Figures 9B,C). A transwell assay was exploited to evaluate migration and invasion in SGC-7901 cells transfected with Si-AMAP1 or Si-NC, and AMAP1 silencing significantly reduced migration and invasion, compared to the controls (Figures 9D–F).

**FIGURE 9:** The effects of knocking out AMAP1on the cell proliferation, migration and invasion. Silence of AMAP1 exhibited lower cell proliferative rate than that in control group as revealed by CCK-8 assay **(A)**. Wound healing test revealed that silence of AMAP1exhibited lower wound healing rate than that in control group **(B,C)**. Transwell assay demonstrated that silence of AMAP1 showed lower migration and invasion ability than that in control group **(D–F)**.

## Discussion

GC is a malignant tumor type with relatively high prevalence, and GC patients with advanced TNM stage typically face unfavorable prognoses (Strong, 2018). Identification of diagnostic and prognostic biomarkers for personalized therapy may help improve the outcome of GC cases. This is the first study to systematically explore the clinical and prognostic value of AMAP1 in GC through analysis of comprehensive bioinformatics in combination with *in vitro* experiments. Both AMAP1 mRNA and protein levels were increased in GC tissues compared to corresponding normal samples. AMAP1 mRNA may thus help differentiate between GC and normal tissues. High AMAP1 mRNA levels were strongly correlated with less favorable clinical characteristics (advanced T, N, and TNM stage) and typically indicated reduced OS and PFS. More importantly, AMAP1 mRNA levels were negatively correlated (*r* = −0.3843; *P* < 0.0001) with has-mir-192 in GC. Our results suggested the diagnostic and prognostic value of AMAP1 in patients with GC, and AMAP1 may be a molecular target in GC treatments.

AMAP1 is an Arf-GTPase-activating protein and regulates local adhesion and actin cytoskeleton remodeling, which are important processes regarding invasion and metastasis of tumor cells (Randazzo et al., 2000; Liu et al., 2002; Muller et al., 2010). AMAP1 overexpression is associated with increased invasion and metastasis of malignant uveal melanoma (Ehlers et al., 2005). Moreover, AMAP1 increases invasion and metastasis of breast cancer cells (Sabe et al., 2009). A different study showed that AMAP1 overexpression promotes invasion of Hep-2 cells (Li et al., 2014). In the current study, integrated genomic analyses revealed that high AMAP1 mRNA levels were significantly correlated with advanced T stage (tumor invasion) and lymph node metastasis in GC patients. However, effects of AMAP1 overexpression and silencing on GC cells require further research.

AMAP1 is an oncogene in various cancers, and high AMAP1 levels predict inferior outcomes in patients with triple-negative breast cancer (He et al., 2020), ovarian cancer (Hou et al., 2014), colorectal cancer (Muller et al., 2010), and laryngeal squamous cell carcinoma (Li et al., 2014). In the current study, we examined for the first time the expression and prognostic value of AMAP1 in GC. Our results demonstrated that AMAP1 mRNA and protein expression were upregulated in GC tissues, compared to adjacent normal tissue, based on the TCGA and HPA databases, which was experimentally confirmed using GC tissue samples and cell lines. Furthermore, GC patients with high AMAP1 mRNA levels showed lower OS and PFS than those with low AMAP1 mRNA levels, as revealed by meta-analyses. Meta-analysis is typically a quantitative synthesis of results of multiple previous studies (Egger et al., 1997); however, this approach may also be used on different datasets. Using meta-analysis, the statistical power of pooled HR was more robust than that of single dataset.

MicroRNAs are small non-coding RNAs of 17–25 nucleotides, which are essential for post-transcriptional regulation gene expression (Shin and Chu, 2014). MicroRNAs are associated with biological processes including cell proliferation, differentiation, metastasis, and apoptosis of GC cells (Hu et al., 2017; Huan et al., 2019; Zhou et al., 2019). In the present study, we showed for the first time that AMAP1 was negatively correlated with miR-192-3p. To our knowledge, this is the first study to explore the clinical role and the prognostic value of miR-192-3p in GC. High miR-192-3p levels were not only associated with early T stage but were also correlated with increased OS in GC patients. Furthermore, both western blotting and RT-PCR revealed low miR-192-3p expression in GC tissues and cells and high expression in normal tissues and GES-1 cells.

KEGG enrichment analysis of genes co-expressed with AMAP1 based on the TCGA-STAD dataset revealed that AMAP1 is associated with cell-cell adhesion through plasma-membrane adhesion molecules, cell-substrate adhesion, focal adhesion, and cell adhesion molecules (Ikeo et al., 2015; Saias et al., 2015). Cell adhesion is crucial for invasion and metastasis of cancer cells. In the first step of cancer metastasis, epithelial-mesenchymal transition of cancer cells requires dissolving cell-cell adhesion (Kawauchi, 2012). A recent study showed that AMAP1 overexpression can promote epithelial to mesenchymal transition through upregulating N-cadherin and decreasing E-cadherin in ovarian cancer cells (Zhang et al., 2018). Hence, based on our results, we propose that AMAP1 may promote invasion and metastasis in GC through downregulation of cell adhesion pathways.

Our conclusions are predominantly derived from bioinformatic analyses. Even though we used paired GC and normal tissue samples as well as GC cell lines to confirm AMAP1 protein and miR-192-3p expression, the effects of miR-192-3p in GC remain unclear, to some extent. Therefore, further research is required to elucidate the regulatory effect of miR-192-3p on AMAP1 mRNA expression in GC cells.

## Conclusion

AMAP1 is a novel oncogene in GC and is negatively correlated with has-mir-192. High AMAP1 expression indicates advanced T, N, and TNM stages. AMAP1 may be a promising diagnostic and prognostic biomarker of GC. Silencing of AMAP1 in GC cells significantly reduced proliferation, migration, and invasion.

## Data Availability Statement

The original contributions presented in the study are included in the article/Supplementary Material, further inquiries can be directed to the corresponding author/s.

## Ethics Statement

This study plan was approved by the Ethics Committee of Renmin Hospital of Wuhan University (No. WDRY2021-K002). The patients/participants provided their written informed consent to participate in this study.

## Author Contributions

WD designed the research. JL and ST performed the research. ST and YG analyzed the data. JL wrote the manuscript. All authors contributed to the article and approved the submitted version.

## Conflict of Interest

The authors declare that the research was conducted in the absence of any commercial or financial relationships that could be construed as a potential conflict of interest.

## Footnotes

1 http://gepia.cancer-pku.cn

2 www.oncomine.org

3 http://xena.ucsc.edu

4 www.kmplot.com

5 www.proteinatlas.org

6 www.linkedomics.org

7 http://www.webgestalt.org/
